The article "Curcumin synergizes with 5-fluorouracil by impairing AMPK/ULK1-dependent autophagy, AKT activity and enhancing apoptosis in colon cancer cells with tumor growth inhibition in xenograft mice" was retracted in 2022. Reasons: lack of ethics approval or compliance; concerns about the data.

# Curcumin synergizes with 5-fluorouracil by impairing AMPK/ULK1-dependent autophagy, AKT activity and enhancing apoptosis in colon cancer cells with tumor growth inhibition in xenograft mice

**DOI:** 10.1186/s13046-017-0661-7

**Published:** 2017-12-22

**Authors:** Pan Zhang, Ze-Lin Lai, Hui-Fen Chen, Min Zhang, An Wang, Tao Jia, Wen-Qin Sun, Xi-Min Zhu, Xiao-Feng Chen, Zheng Zhao, Jun Zhang

**Affiliations:** 1 Key Laboratory of Brain Functional Genomics (East China Normal University), Ministry of Education, School of Life Sciences, East China Normal University, Shanghai, 200062 China; 2 Department of Clinical Laboratory, Shanghai First Maternity and Infant Hospital, Tongji University School of Medicine, Shanghai, 201204 China; 3 Department of Clinical Laboratory, Shanghai Public Health Clinical Center Affiliated to Fudan University, Shanghai, 201508 China; 4 Department of Thoracic Surgery, Huashan Hospital, Fudan University, Shanghai, 200040 China; 5 INSERM-UGA U1209, CNRS UMR5309, Institute for Advanced Biosciences, F-38700 La Tronche, France

**Keywords:** Curcumin, 5-fluorouracil, Autophagy, Colon cancer, Combination chemotherapy

## Abstract

**Background:**

Chemoresistance is a major obstacle that limits the benefits of 5-Fluorouracil (5-Fu)-based chemotherapy for colon cancer patients. Autophagy is an important cellular mechanism underlying chemoresistance. Recent research advances have given new insights into the use of natural bioactive compounds to overcome chemoresistance in colon cancer chemotherapy. As one of the multitargeted and safer phytomedicines, curcumin has been reported to work as cancer-specific chemosensitizer, presumably via induction of autophagic signaling pathways. The precise therapeutic effect of curcumin on autophagy in determining tumorous cells’ fate, however, remains unclear. This study was conducted to investigate the differential modulations of the treatments either with 5-Fu alone or 5-Fu combined with curcumin on cellular autophagic responses and viabilities in the human colon cancer cells HCT116 and HT29, and explore molecular signaling transductions underlying the curcumin-mediated autophagic changes and potentiation of 5-Fu’s cytotoxicity in vitro and in vivo.

**Methods:**

Cell proliferation assay and morphology observation were used to identify the cytotoxicity of different combinations of curcumin and 5-Fu in HCT116 and HT29 cells. Cell immunofluorescence assay, Flow cytometry and Western blot were employed to detect changes of autophagy and the autophagy-related signaling pathways in the colon cancer cells and/or xenograft mice.

**Results:**

Curcumin could significantly augment the cytotoxicity of 5-Fu to the tumorous cells, and the pre-treatment with curcumin followed by 5-Fu (pre-Cur) proved to be the most effective one compared to other two combinations. The chemosensitizing role of curcumin might attribute to the autophagy turnover from being activated in 5-Fu mono-treatment to being inhibited in the pre-Cur treatment as indicated by the changes in expression of beclin-1, p62 and LC3II/LC3I and the intensity of Cyto-ID Green staining. The autophagic alterations appeared to be contributed by down-regulation of not only the phospho-Akt and phospho-mTOR expressions but the phospho-AMPK and phospho-ULK1 levels as well. The cellular activation of AMPK by addition of A-769662 to the pre-Cur combination resulted in reversed changes in expressions of the autophagy protein markers and apoptotic status compared to those of the pre-Cur combination treatment. The findings were validated in the xenograft mice, in which the tumor growth was significantly suppressed in the mice with 25-day combination treatment, and meanwhile expressions of the autophagy markers, P-AMPK and P-ULK1 were all reversely altered in line with those observed in HCT116 cells.

The article "Curcumin synergizes with 5-fluorouracil by impairing AMPK/ULK1-dependent autophagy, AKT activity and enhancing apoptosis in colon cancer cells with tumor growth inhibition in xenograft mice" was retracted in 2022. Reasons: lack of ethics approval or compliance; concerns about the data.

**Conclusion:**

Pre-treatment with curcumin followed by 5-Fu may mediate autophagy turnover both in vitro and in vivo via AMPK/ULK1-dependent autophagy inhibition and AKT modulation, which may account for the increased susceptibility of the colon cancer cells/xenograft to the cytotoxicity of 5-Fu.

**Electronic supplementary material:**

The online version of this article (10.1186/s13046-017-0661-7) contains supplementary material, which is available to authorized users.

## Background

Colon cancer is one of the most common malignancies in human worldwide [1]. 5-Fluorouracil (5-Fu), a fluoropyrimidine analog, is chemotherapeutic agent widely used for the treatment of this cancer type [2]. While the non-specific cytotoxicity narrows its clinical therapeutic index with small differences between therapeutic and toxic doses, therapeutic resistance of 5-Fu is often occurred and results in poor outcome for the patients [3]. Although the combinational use of 5-Fu with other agents such as oxaliplatin, irinotecan or bevacizumabhas has significantly improved the prognosis and clinical benefits [4, 5], there remains a critical need for better understanding of molecular basis that accounts for the chemotherapeutic resistance, and hereby to uncover novel therapeutic strategies for extending survival while decreasing resistance and increasing therapeutic window in colon cancer patients.

Cancer cells trigger multiple signaling to escape from the cytotoxicity of chemotherapeutics. Autophagy, as a route of programmed cell death, has been increasingly studied in cancer therapy [6], and is thought to contribute to autophagic cell death via lysosomes-related cell degradation [7]. On the other hand, autophagy could promote tumor progression by providing metabolic fuel for cell survival when encountered environmental stressors such as nutrient starvation, hypoxia or treatment with chemotherapeutic agents [8–10]. Such a “double-edged sword” role of autophagy in cancer is dependent on tumor cell types and their specific microenvironment. Nevertheless, evidence has been accumulated in support of the notion that autophagy could be an important cellular mechanism towards chemoresistance in various malignancies [11, 12]. Modulation of autophagy could be therefore a promising new strategy to overcome chemoresistance in cancer therapy.

The article "Curcumin synergizes with 5-fluorouracil by impairing AMPK/ULK1-dependent autophagy, AKT activity and enhancing apoptosis in colon cancer cells with tumor growth inhibition in xenograft mice" was retracted in 2022. Reasons: lack of ethics approval or compliance; concerns about the data.

Curcumin is well-known to be the main active component responsible for the majority of the medicinal properties of turmeric. In addition to otherwise described, curcumin has increasingly attracted scientific and clinical interests due to its wide spectrum of pharmacological activities upon multiple biological targets in preventing tumor initiation, progression, and dissemination in a number of human cancers [13, 14]. Moreover, the neglectable toxicity makes curcumin a very suitable adjuvant in disease, including cancer treatment [15]. Indeed, curcumin could act as cancer-specific chemosensitizer, presumably via induction of autophagic signaling pathways [16]. To the context of gaining insights into novel therapeutic strategies, however, the precise therapeutic effect of curcumin, especially under circumstance of chemo-related resistance, on autophagy in determining tumorous cells’ fate remains unclear. Thus, this study was designed to investigate the differential modulations of the treatments either with 5-Fu alone or 5-Fu combined with curcumin on cellular autophagic responses and viabilities in the human colon cancer cells HCT116 and HT29, and then to further explore if such autophagic responses could be attributed to curcumin-mediated changes on Akt/mTOR/ULK1 and AMPK-ULK1 signal transductions and hereby potentiate 5-Fu’s cytotoxicity in vitro and in vivo.

## Methods

### Chemicals and cell culture

The colon cancer cell lines HCT116 and HT29 were purchased from Cell Bank of the Chinese Academy of Sciences (Shanghai, China). Cells were cultured in RPMI-1640 medium (HyClone) with 10% fetal bovine serum (Gibco), 50 μg/mL streptomycin and 50 IU/mL penicillin, and were maintained at 37 °C in a humidified incubator containing 5% CO_2_. 100 mM Stock solutions of 5-Fu (Sigma) and curcumin (Sigma), and 10 mM stock solutions of A-769662 (Selleck) were prepared in dimethylsulfoxide (DMSO) (Sigma), respectively.

The article "Curcumin synergizes with 5-fluorouracil by impairing AMPK/ULK1-dependent autophagy, AKT activity and enhancing apoptosis in colon cancer cells with tumor growth inhibition in xenograft mice" was retracted in 2022. Reasons: lack of ethics approval or compliance; concerns about the data.

### Cell proliferation assay and morphology observation

Cells were mono-treated with 5-Fu or curcumin for 24 h or 48 h, and co-treated with 5-Fu and curcumin in different combinations basing on their concentrations and treatment time points. Cell proliferation was examined using the Cell Counting Kit-8 (CCK-8) (Beyotime), according to the manufacturer’s protocols. The cell morphology was observed using a TE2000-S fluorescence microscope (Nikon).

### Cell immunofluorescence assay

Autophagic response in different cell groups treated with 5-Fu alone or 5-Fu combined with curcumin was determined using the Cyto-ID Autophagy Detection Kit (ENZO), according to the procedures provided by the manufacturer. Briefly, after treatments with the testing agents, the culture medium in each well was removed. The cell residues were washed twice with the assay buffer, and 100 μl of Dual Detection Reagent (2 μl of Cyto-ID Green Detection Reagent and 1 μl of Hoechst 33,342 Nuclear Stain in 1 mL of cell culture medium) was then dispensed in each well. The cells were protected from light and incubated at 37°C for 30 min. After washing again as above, the cell samples were analyzed using the fluorescence microscope.

The apoptotic response at single cell level in different cell groups was determined quantitatively using the In Situ Cell Death Detection Kit (Roche), according to the procedures provided by the manufacturer. Briefly, after treatment with the testing agents, the cell samples were air-dried and fixed with freshly prepared 4% paraformaldehyde in PBS (pH 7.4) for 1 h at room temperature, followed by rinsing with PBS and incubating on ice for 2 min in freshly prepared 0.1% Triton X-100 in 0.1% sodium citrate. With addition of 50 μl of TUNEL reaction mixtures to each well, the samples were incubated at 37°C in dark for 60 min under a humidified atmosphere. After rinsing, the samples were observed using the fluorescence microscope.

### Flow cytometry

Pretreated with curcumin (0, 10, 20, 30 μM) and then 20 μM 5-Fu, the cells were collected by trypsinization and the cell density was kept at 3 × 10^5^ cells per ml. The cell samples were washed twice via centrifugation at 1200 rpm and resuspended in 0.5 ml of freshly diluted Cyto-ID Green Detection Reagent (1 μl Cyto-ID Green Detection Reagent to a final volume of 2 ml with cell culture medium). After 30 min incubation at 37°C in the dark, the samples were analyzed in the green (FL1) channel of flow cytometer.

### Western blot

The whole proteins in each cell samples were extracted by RIPA Lysis Buffer containing 1 mM PMSF (Beyotime). The protein was blocked and incubated with the primary antibodies against beclin-1, p62/SQSTM1 and LC3 (MBL; 1:1000), caspase 3, GAPDH, P-Akt (Ser473), P-AMPK (Thr172), P-ULK1 (Ser317) and P-mTOR (Ser2448) (Cell Signaling; 1:1000), overnight at 4 °C, respectively. The protein was then incubated with HRP-conjugated secondary antibody (1:5000) for 1 h at room temperature. The protein was detected using the eECL Western Blot Kit (Beyotime).

The article "Curcumin synergizes with 5-fluorouracil by impairing AMPK/ULK1-dependent autophagy, AKT activity and enhancing apoptosis in colon cancer cells with tumor growth inhibition in xenograft mice" was retracted in 2022. Reasons: lack of ethics approval or compliance; concerns about the data.

### Tumor suppression experiment in vivo

Thirty male BALB/c-nu/nu mice purchased from Shanghai SIPPR-BK Laboratory Animal Company, four-week-old and about 18-22 g, were housed on 12/12 h light/dark cycles with ad libitum access to rat chow and water. They were allowed to acclimatize for 1 week prior to treatment. For treatments, HCT116 cells (2 × 10^6^) in 0.2 ml PBS or saline was injected into the right flank of test mice to form xenograft tumors and the mice were divided into five groups when they developed the tumor in similar size: normal group (no tumor in mice), control group (with tumor and intraperitoneal injection of equivalent solvent), cur group (with tumor and intraperitoneal injection of curcumin every day), 5-Fu group (with tumor and intraperitoneal injection of 5-Fu every other day) and Pre-cur group (with tumor and intraperitoneal injection of curcumin every day followed by 5-Fu every other day). Curcumin (40 mg/kg) and 5-Fu (30 mg/kg) were dissolved in 0.9% NaCl solution with 10% Tween 80 and 1% DMSO. The tumor volume was measured as *v* = 1/2*ab* ^2^, where a is the longer axis diameter and b the shorter axis diameter. The tumor volume was measured every 5 days and food intake was measured every 3 days.

### Data analysis

Three or more independent experiments were performed for WST viability assay, western blot, immunofluorescent images, TUNEL assay and flow cytometry analysis. The values were expressed as the mean ± SE. The statistical significance of the mean values among different groups was determined using one-way ANOVA, followed Student’s *t*-test.

## Results

### Curcumin augments cytotoxicity of 5-fu in HCT116 and HT29 cells

The concentration (0, 10, 20, 40, 60, 80, 100 and 120 μM)- and time (24 and 48 h)-related effects of mono-treatment of 5-Fu or curcumin on the viabilities of HCT116 and HT29 were evaluated. Both testing agents displayed a weaker inhibitory effect, respectively, on the cell lines, although the inhibitory ratios for 48 h treatments were higher than those for 24 h (Fig. 1a, Additional file 1: Figure S1A). The role of 5-Fu alone was increased within a lower concentration range (i.e., <40 μM), but became plateaued beyond 40 μM, suggesting a possible resistance of 5-Fu in the cancer cells (Fig. 1a, Additional file 1: Figure S1A). Such a cellular behavior of 5-Fu was distinguishable from that of curcumin, in which an increasing trend of inhibitory role of curcumin appeared to cover the whole range of the testing concentrations (Fig. 1a, Additional file 1: Figure S1A). The weak cytotoxicity of 5-Fu against the HCT116 cells, especially when used at low concentration (20 μM) and for short time (24 h), was also morphologically confirmed as illustrated in Additional file 2: Figure S2A. Subsequently, the inhibitory effects of different combination treatments, with low exposure concentrations (10 and 20 μM) and time (24 h), of 5-Fu and curcumin in HCT116 and HT29 were examined (Fig. 1b, Additional file 1: Figure S1B). With initial comparisons for optimal inhibitory efficacy of different combination protocols, i.e., pretreatment with curcumin and then 5-Fu (pre-Cur), treatment with 5-Fu and curcumin at the same time (5-Fu + Cur), and pretreatment with 5-Fu and then curcumin (pre-5-Fu), the pre-Cur (both agents were 20 μM) was found to be the best as its inhibitory ratio was over 50% in HCT116 cells (Fig. 1b-d), indicating that pretreatment with 20 μM curcumin could significantly augment the cytotoxicity of 20 μM 5-Fu against the cancer cells as compared with that of 5-Fu alone (Additional file 2: Figure S2B). This protocol, i.e., the pre-Cur (both agents were 20 μM), was therefore used in subsequent experiments except as otherwise specified.

The article "Curcumin synergizes with 5-fluorouracil by impairing AMPK/ULK1-dependent autophagy, AKT activity and enhancing apoptosis in colon cancer cells with tumor growth inhibition in xenograft mice" was retracted in 2022. Reasons: lack of ethics approval or compliance; concerns about the data.

**Fig. 1:** Viability of colon cancer HCT116 cells treated with 5-Fu or curcumin, alone or in different combinations. **a**. Growth-inhibitory curves of HCT116 cells exposing to gradient concentrations of 5-Fu or curcumin alone: (a) and (b) for 24 h, and (c) and (d) 48 h, respectively. **b**. Comparison of viabilities in HCT116 treated for 48 h with different combinational protocols. Cur: curcumin alone, 5-Fu: 5-Fu alone, pre-Cur: pretreated with curcumin for 24 h followed by 5-Fu for 24 h, Cur + 5-Fu: co-treated with 5-Fu and curcumin for 24 h, pre-5-Fu: pretreated with 5-Fu for 24 h followed by curcumin for 24 h.: (a) 10 μM curcumin/10 μM 5-Fu, (b) 10 μM curcumin/20 μM 5-Fu, (c) 20 μM curcumin/10 μM 5-Fu and (d) 20 μM curcumin and 20 μM 5-Fu

### Cellular autophagic turnover by the combination treatment accounts for increased cytotoxicity of 5-fu in HCT116 and HT29 cells

To address cellular mechanisms underlying the alterations in cytotoxicity of 5-Fu mentioned above, the autophagic responses following 5-Fu alone or the combination treatments in the tumorous cells were examined. The cell immunofluorescence staining showed enhanced Cyto-ID Green signals in HCT116 cells treated with 5-Fu alone (Fig. 2a). In consistent with this, 5-Fu mono-treatment suppressed p62 and activated beclin-1 expressions, while also caused LC3I to LC3II transformation (Fig. 2b, Additional file 3: Figure S3). By contrast, the combination treatments (pre-Cur) obviously weakened the Cyto-ID Green signals in the cells (Fig. 3a and b), and reversed the changes brought by 5-Fu alone in the expressions of p62 and beclin-1 and the transformation of LC3I to LC3II (Fig. 3c, Additional file 4: Figure S4A). The results revealed a curcumin-mediated autophagy inhibition underlying, at least in part, the increased cytotoxicity of 5-Fu in the colon cancer cells.

The article "Curcumin synergizes with 5-fluorouracil by impairing AMPK/ULK1-dependent autophagy, AKT activity and enhancing apoptosis in colon cancer cells with tumor growth inhibition in xenograft mice" was retracted in 2022. Reasons: lack of ethics approval or compliance; concerns about the data.

**Fig. 2:** Immunofluorescent images of HCT116 cells treated with or without 5-Fu. **a**. Hoechst 33,342 staining (blue) indicates nucleus and Cyto-ID Green staining (green) autophagy status. **b**. Western blot analysis of beclin-1, p62 and LC3II/LC3I in HCT116 cells after exposing to varied concentrations of 5-Fu for 24 h. *, *p* < 0.05, and **, *p* < 0.01, compared to the vehicle (0 μM 5-Fu) cell group

**Fig. 3:** Cellular autophagic turnover by combinational treatment of 5-Fu and curcumin. **a**. Immunofluorescent images of HCT116 and HT29 cells treated with the pre-Cur protocol. Hoechst 33,342 staining (blue) indicates nucleus and Cyto-ID Green staining (green) autophagy status. **b**. Flow cytometry analysis of autophagy in HCT116 cells pretreated with varied concentrations of curcumin for 24 h and then 20 μM of 5-Fu for 24 h. The percentage value indicates the proportion of autophagy-positive cells, detected as an increase in the number of FITC (FL-1)-labeled cells. **c**. Western blot analysis of beclin-1, p62 and LC3II/LC3I in HCT116 cells pretreated with varied concentrations of curcumin for 24 h and then 20 μM of 5-Fu for 24 h. *, *p* < 0.05, and **, *p* < 0.01, compared to the vehicle (0 μM curcumin) cell group

### Molecular alteration in AMPK/ULK1 signaling accounts for the autophagy inhibition in HCT116 and HT29 cells

To address molecular signaling pathway underlying the curcumin-modulated autophagic turnover, changes in the autophagy trigger ULK1 and its upstream effectors, AMPK and Akt/mTOR, following varied concentrations of 5-Fu alone or of the combination treatments were examined. Mono-treatment of 5-Fu appeared to reduce the levels of P-Akt and P-mTOR and to increase the levels of P-ULK1, though with no apparent dose-dependency, while had no effect on the levels of P-AMPK (Fig. 4a). In contrast, the combination treatment appeared to down-regulate not only the P-Akt and P-mTOR expressions but also the P-AMPK and P-ULK1 levels in a curcumin concentration-related manner (Fig. 4b, Additional file 4: Figure S4B), suggesting that alterations in AMPK/ULK1 signaling are responsible for the changes in autophagic status in HCT116 and HT29.

The article "Curcumin synergizes with 5-fluorouracil by impairing AMPK/ULK1-dependent autophagy, AKT activity and enhancing apoptosis in colon cancer cells with tumor growth inhibition in xenograft mice" was retracted in 2022. Reasons: lack of ethics approval or compliance; concerns about the data.

**Fig. 4:** Analysis of P-Akt, P-mTOR, P-AMPK and P-ULK1 expression levels in HCT116 cells. **a**. Treatment for 24 h by varied concentrations of 5-Fu alone. **b**. The pre-Cur treatment (varied concentrations of curcumin and 20 μM 5-Fu). *, *p* < 0.05, **, *p* < 0.01, and ***, *p* < 0.001, compared to the vehicle (0 μM 5-Fu or 0 μM curcumin) cell group

### Curcumin sensitizes colon cancer cells to 5-fu via inhibition of AMPK-modulated autophagy pathway

To further dissect the essentiality of AMPK in curcumin-mediated autophagy inhibition that led to enhanced susceptibility of the cancer cells to 5-Fu, the cellular autophagic changes as well as the apoptotic status in HCT116 cells were examined following the combination treatment with addition of A-769662, a selective AMPK activator. The results demonstrated that changes in the expressions of p62 and beclin-1, the transformation of LC3I to LC3II, and the intensity of Cyto-ID Green staining were all neutralized as compared with those of the pre-Cur treatment (Fig. 5a and b). In line with this, the apoptotic effect of the pre-Cur treatment was also counteracted in response to the addition of A-769662 as indicated by WST analysis, TUNEL analysis and the changes of caspase 3 (Fig. 5c and d, Additional file 5: Figure S5).

**Fig. 5:** Effects of A-769662 added to the pre-Cur on autophagic and apoptotic status in HCT116 cells. **a**. Immunofluorescent images. Hoechst 33,342 staining (blue) indicates nucleus and Cyto-ID Green staining (green) autophagy status. **b**. Western blot analysis of beclin-1, p62 and LC3II/LC3I. **c**. Comparison of viability of colon cancer HCT116 cells. **d**. Western blots analysis of cleaved-caspase-3. *, *p* < 0.05, **, *p* < 0.01, and ***, *p* < 0.001

### Increased anti-tumor effect of the combination treatment is accompanied by AMPK/ULK1-dependent autophagic turnover in vivo in subcutaneous xenograft mice

To verify the cellular and molecular findings described above, the therapeutic efficacies in terms of the tumor size as well as autophagic status were examined in the tumor xenograft mice. The results demonstrated that the growth of tumor was significantly suppressed in mice with 25-day combination treatment of curcumin (40 mg/kg) and 5-Fu (30 mg/kg) as compared with those in the controls as well as in mice with mono-curcumin (40 mg/kg) or mono-5-Fu (30 mg/kg) treatment (Fig. 6a). Correspondingly, the expressions of p62, beclin-1, LC3II/LC3I ratio, P-AMPK and P-ULK1 were all reversely altered in line with the changes of these proteins as observed in vitro in HCT116 cells, pinpointing an AMPK/ULK1-mediated autophagy inhibition in tumor tissues of the mice with the combination treatment (Fig. 6b). Moreover, the food-intake of the tumor-bearing mice were less impacted by the combination treatment as compared with those by the 5-Fu mono-treatment (Fig. 6c), suggesting that curcumin, when used as an adjuvant agent, could not only increase the anti-tumor efficacy, but also somehow relieve appetite-related side-effect, of 5-Fu.

The article "Curcumin synergizes with 5-fluorouracil by impairing AMPK/ULK1-dependent autophagy, AKT activity and enhancing apoptosis in colon cancer cells with tumor growth inhibition in xenograft mice" was retracted in 2022. Reasons: lack of ethics approval or compliance; concerns about the data.

**Fig. 6:** Analysis of anti-tumor effect of combination treatment of 5-Fu (30 mg/kg) and curcumin (40 mg/kg) and AMPK/ULK1-related autophagy in subcutaneous xenograft mice. **a**. Photographs of nude mice bearing HCT116-deliveried tumors after 25-day treatment. The tumor volume was measured using Vernier calipers and calculated as described in Materials and Methods. **b**. Western blots analysis of beclin-1, p62, LC3II/LC3I, P-AMPK and P-ULK1 expression levels in tumorous tissue of the mice. **c**. The change of food intake of the xenograft mice during the 25-day treatment. *, *p* < 0.05, and **, *p* < 0.01

## Discussion

Serious toxicity/side-effect and therapeutic resistance are considered to be two major obstacles for a successful cancer chemotherapy translated from bench to bed [17]. This may be due to the scarce knowledge of cancer cell signaling network and bypass mechanisms. As an effort among others that deserves attention, a novel combinational strategy with aims to reverse chemoresistance has recently been proposed, in which an adjuvant drug is sequentially added to target resistance caused by major chemotherapy [18]. The present study demonstrates a unique combination of curcumin and 5-Fu, which though has been previously documented [19], to assess if and how curcumin could enhance the anti-cancer efficacy of 5-Fu in human colon cancer cells.

It is well-known that curcumin is efficient and safe for the prevention and treatment of varied pathological conditions, including cancer [20], despite its clinical benefits of curcumin are still limited due to its poor pharmacokinetic properties and bioavailability in vivo [21]. Given the fact that curcumin induces apoptosis via pleiotropic mechanisms in various cancer types [20, 22], several studies demonstrated the high interest of using curcumin as potent chemosensitizer to improve the therapeutic effects of cisplatin, mitomycin C, γ-Radiation, and other chemotherapeutics [23–25]. Particularly, co-treatment of curcumin and 5-Fu, both at a single dose-level, promoted chemosensitivity in colon carcinoma cells [26]. In the present study, with initial observations of 5-Fu-resistance in HCT116 and HT29 cells (Fig. 1a, Additional file 1: Figure S1A), we investigated the differential sensitizing effects of curcumin on the cytotoxicity of 5-Fu by taking three different combinations, i.e., pre-treatment of curcumin followed by 5-Fu (pre-Cur), co-treatment of two agents (5-Fu + Cur) and post-treatment of curcumin following 5-Fu (pre-5-Fu). The cellular viability data showed that the pre-Cur was the most effective regimen compared to others (Fig. 1b, Additional file 1: Figure S1B), and that curcumin pretreatment at 20μM could significantly sensitize the anti-tumor activity of 5-Fu at a lower dosage (20μM), as compared with that of 5-Fu alone (Fig. 1b-d, Additional file 1: Figure S1B–d). Similarly, in the HCT116-derived xenograft mouse model, we further found that pretreatment of curcumin followed by a lower dosage of 5-Fu (30 mg/kg) exhibited not only a significant reduction of the tumor size but also an improvement in food-intake status, which was absent in mono-treatment groups (Fig. 6a and c). Nevertheless, our findings, from both in vitro and in vivo assays, provide valuable insights into the novel benefits of curcumin on increasing chemosensitization and decreasing undesirable toxicity, whatever being contained in a regular diet or as an adjuvant medicine, for long-term use in patients with colon cancer prior to or during 5-Fu-based chemotherapy.

The article "Curcumin synergizes with 5-fluorouracil by impairing AMPK/ULK1-dependent autophagy, AKT activity and enhancing apoptosis in colon cancer cells with tumor growth inhibition in xenograft mice" was retracted in 2022. Reasons: lack of ethics approval or compliance; concerns about the data.

Autophagy is an evolutionarily conserved catabolic process with essential functions in cellular homeostasis and cell survival under both physiological and pathological conditions [27]. In addition to its housekeeping roles in removing damaged DNA, dysfunctional proteins and defective organelles, autophagy also involves in tumorigenesis and cancer cell metabolism [28, 29]. Here, we proved that the dysregulation of autophagy also contributes to reduced cytotoxicity of 5-Fu. To understand synergistic effects of curcumin with 5-Fu, we compared the effects of 5-Fu alone with that of pre-Cur on cells’ autophagic process by immunofluorescence Cyto-ID Green staining and Western blotting of the autophagic proteins p62, beclin-1 and LC3II/LC3I. We showed that 20 μM 5-Fu activated autophagy after 24 h (Fig. 2, Additional file 3: Figure S3), which was reserved by pre-Cur combinational treatment (Fig. 3, Additional file 4: Figure S4-A). In contrast to our findings, Yao et al. reported that 140 mM 5-Fu reduced autophagy in SNUC5 colon cancer cells after more than 6 months treatment [30]. While another recent study, in concert with that of us, demonstrated that autophagy inhibitor 3-MA could potent 25 μM 5-Fu’s cytotoxicity in HT29 colon cancer cells after 48 h treatment [31]. The discrepancies between seemingly different impacts of 5-Fu on autophagy would be explained by the differences on its using dosages, times, as well as the different context with different colorectal cancer cell types [32, 33]. On the other hand, from the pathophysiological view of autophagy, which is generally regarded as a cellular adaptation mechanism to counteract cellular stress, for example in chemotherapy, that would trigger pro-survival signals escaping from apoptosis or cell death [34, 35], the 5-Fu-triggered autophagy activation in our experiments may be a survival response of the colon cancer cells to the cytotoxic stimulus of 5-Fu. In addition to 5-Fu, curcumin has also been believed to be an autophagy regulator associated with its anti-cancer activity, for instance as an autophagy inducer in human gastric cancer cells [36], human melanoma cells [37], osteosarcoma MG63 cells [38] and HCT116 colon cancer cell line [39], and as a blocker in malignant mesothelioma cells [40]. The molecular changes underlying curcumin-mediated autophagic responses were also documented for cutaneous T-cell lymphoma to be relevant to the degradation of beclin-1, which is a component of class III phosphatidylinositol 3-kinase (IIIPI3K) and has an up-regulating effect on autophagosome [41], and thereby the accumulation of microtubule-associated protein-1 light chain 3 (LC3I), which promotes the death of the cancer cells [42]. To our knowledge, there is no report addressing the critical role of the combinational use of curcumin with 5-Fu in autophagic regulation that promotes chemosensitization in the colon cancer cells. Collectively, 5-Fu-induced activation of autophagy might suggest a cellular mechanism responsible for, at least in part, the low susceptibility of HCT116 and HT29 colon cancer cells to 5-Fu mono-treatment, and the cellular autophagic turnover we observed following the pre-Cur combinational treatment might thus further reveal an autophagy inhibitory mechanism underlying, at least partially, the increased cytotoxicity of 5-Fu when curcumin actioned as an autophagy inhibitor.

The article "Curcumin synergizes with 5-fluorouracil by impairing AMPK/ULK1-dependent autophagy, AKT activity and enhancing apoptosis in colon cancer cells with tumor growth inhibition in xenograft mice" was retracted in 2022. Reasons: lack of ethics approval or compliance; concerns about the data.

Given the fact that curcumin’s pleiotropic activity on cancer prevention [2–4], several earlier studies have further illustrated this interest of combinational using of curcumin with 5-Fu, by showing its sensitizing effect against 5-Fu resistance in varied cancer cell types such as human gastric cancer cells through inhibition of the NFκB survival-signaling pathway [43], or particularly in different sub-types of colon cancer cell lines, via miRNA-induced suppression of epithelial-to-mesenchymal transition [26], or the modulation of EGFR and IGF-1R. [19] With attempt to explore molecular interactions underlying the autophagic responses following 5-Fu mono-treatment and the pre-Cur combinational treatment, we investigated the changes within the core autophagy machinery including the autophagic trigger ULK1 and its upstream effectors Akt, mTOR and AMPK. It is generally believed that AMPK activation could dampen mTOR expression and thereby trigger autophagy via phosphorylation of ULK1. Accumulated evidence has indicated that under different nutritional statuses AMPK is coordinated closely with mTOR in regulating autophagy through direct phosphorylation of ULK1, mainly at site Ser317 and/or Ser777 within the Ser/Thr-rich domain [44, 45]. For instance, under basal condition, activated Akt/mTOR signaling is able to inhibit autophagy by disrupting the AMPK-ULK1 interaction, whereas during nutrient deficiency AMPK could promote autophagy by direct activation of ULK1, presumably at site Ser317 and /or Ser777 [45]. Although these studies has proposed a direct connection between nutrient-sensing kinases and autophagic activation, the further challenge still remains as to if these are other signaling pathways, such as feedback signals, that could even more criticaly regulate and control autophagy, as autophagy itself is such a “double-edged sword” process and requires to be precisely regulated [46]. Our data indicate that mono-5-Fu-activated autophagy in HCT116 and HT29 cells (Fig. 2, Additional file 3: Figure S3) appeared to be caused by the blockage of phosphorylation of Akt/mTOR and thereby activation of P-ULK1(Ser317), though no obvious changes found for AMPK signaling (Fig. 4a), whereas the pre-Cur combinational treatment appeared to down-regulate not only the P-Akt and P-mTOR expressions but also the P-AMPK and P-ULK1(S317) levels (Fig. 4b, Additional file 4: Figure S4-B). Although the question to these results still remains as to why under the circumstance of 5-Fu mono-treatment, ULK1(Ser317)-mediated activation of autophagy was apparently responsible for the inhibition of Akt/mTOR signaling pathway but not activation of AMPK, our data imply a functional substrate (ULK1Ser317)-competitive interaction between Akt/mTOR/ULK1 and AMPK/ULK1 pathways in favor of the latter that eventually leads to the autophagy reversal from being activated in response to 5-Fu alone to being inhibited in response to the pre-Cur treatment (Figs. 2 and 3, Additional file 3: Figure S3 and Additional file 4: Figure S4). Moreover, PI3K signaling takes vital role in tumor initiation and progression, and the signaling pathway is also genetically altered in numerous cancer types, including the tumor of colon, which was detected with high frequency of PIK3CA activating mutation as well as relative lower frequency of PTEN inactivating mutation [47]. PIK3CA and PTEN mutations both direct PI3K tumorigenesis largely through mediating Akt activity. And we selected two PIK3CA activating mutation cells HCT116 and HT29 to study the anti-tumor efficiency of different treatments either with 5-Fu alone or 5-Fu plus curcumin, so it is of interest to compare their impacts on Akt. As mentioned above, curcumin potentiated the inhibition of Akt by 5-Fu in a dose-dependent manner in HCT116 cells (Fig. 4b). In contrast, the treatment of 5-Fu alone only showed mild and seemingly transient Akt inhibition, which is absent at high dosages of 5-Fu (Fig. 4a), implying that curcumin not only functions as an inhibitor of autophagy to synergize the cytotoxicity of 5-Fu in colon cancer cells, but also works as a cytotoxicity enhancer via directly inhibition of Akt activity. Furthermore, curcumin-mediated AMPK-dependent autophagic turnover towards sensitization of HCT116 cells to 5-Fu was oppositely confirmed by addition of A-769662, a selective agonist of AMPK, to the pre-Cur treatment, in which the A-769662-activated AMPK led to an autophagic reverse as evidenced by the increased levels of both beclin-1 and the ratio of LC3II/LC3I and an decreased expression of p62 (Fig. 5b), and by the elevated intensity of Cyto-ID Green Staining (Fig. 5a) as compared with those found in the pre-Cur treatment, and consequently resulting in a reduced apoptosis and inactivation of caspase 3 (Fig. 5c and d, Additional file 5: Figure S5). More importantly, all these cellular and molecular findings could be well translated into in vivo anti-tumor outcomes as shown by the measures of tumor-size and food-intake for the HCT116-delivered xenograft mice following the 25-day combination treatment of curcumin (40 mg/kg) and 5-Fu (30 mg/kg) (Fig. 6a and c). Correspondingly, an AMPK/ULK1-regulated autophagic mechanism underlying the tumor-suppression efficacies of the combinational therapeutics in the tumor-bearing mice was also evident (Fig. 6b). Taking together, our in vitro and in vivo studies provide novel information regarding to 5-Fu’s lower therapeutic index and the underlying cellular and molecular mechanisms, as well as potential use of curcumin as an autophagy inhibitor to synergize with 5-Fu’s anti-tumor effects.

The article "Curcumin synergizes with 5-fluorouracil by impairing AMPK/ULK1-dependent autophagy, AKT activity and enhancing apoptosis in colon cancer cells with tumor growth inhibition in xenograft mice" was retracted in 2022. Reasons: lack of ethics approval or compliance; concerns about the data.

In summary, we show that autophagy was activated by mono-treatment of 5-Fu in vitro in the human colon carcinoma HCT116 and HT29 cell lines and in vivo in tumor tissues of the xenograft mice. This autophagy activation was found to predispose insensitivity of the tumor cells to 5-Fu. Pre-treatment with curcumin followed by 5-Fu (combination treatment), however, caused autophagy turnover both in vitro and in vivo, which was found to contribute to increased susceptibility of the colon cancer cells/xenograft to the anti-proliferative/anti-growth activities of 5-Fu.

## Conclusions

Our results suggest, as illustrated in Fig. 7, that additive using of curcumin could amplify 5-Fu anti-tumor effects through suppression of Akt signaling and autophagic activity via damping AMPK/ULK1 signaling.

**Fig. 7:** Proposed mechanistic signaling pathways in the colon cancer cells of Akt/mTOR/ULK1(Ser317) autophagy activation in response to 5-Fu alone (**a**), and of AMPK/ULK1(Ser317) autophagy inhibition in response to the combination of 5-Fu and curcumin (**b**)

## Additional files

Additional file 1: Figure S1. Viability of colon cancer HT29 cells treated with 5-Fu or curcumin, alone or in different combinations. A. Growth-inhibitory curves of HT29 cells exposing to gradient concentrations of 5-Fu or curcumin alone: (a) and (b) for 24 h, and (c) and (d) 48 h, respectively. B. Comparison of viabilities in HT29 cells treated for 48 h with different combinational protocols. Cur: curcumin alone, 5-Fu: 5-Fu alone, Pre-Cur: pretreated with curcumin for 24 h followed by 5-Fu for 24 h, Cur + 5-Fu: co-treated with 5-Fu and curcumin for 24 h, Pre-5-Fu: pretreated with 5-Fu for 24 h followed by curcumin for 24 h: (a) 10 μM curcumin/10 μM 5-Fu, (b) 10 μM curcumin/20 μM 5-Fu, (c) 20 μM curcumin/10 μM 5-Fu and (d) 20 μM curcumin and 20 μM 5-Fu. (PDF 148 kb)

Additional file 2: Figure S2. Images of colon carcinoma cells HCT116. (A) HCT116 cells were treated with 5-Fu for 24 h and 48 h, respectively. (B) HCT116 cells were treated with solvent for 48, pretreated with solvent for 24 h and then 20 μM 5-Fu for 24 h, pretreated with 20 μM Cur for 24 h and then 20 μM 5-Fu for 24 h, respectively. (PDF 441 kb)

Additional file 3: Figure S3. Western blot analysis of p62 and LC3 II/I in HT29 cells after exposing to varied concentrations of 5-Fu for 24 h. *, *p* < 0.05 and **, *p* < 0.01 compared to the vehicle (0 μM 5-Fu) cell group. (PDF 186 kb)

Additional file 4: Figure S4. Western blot analysis of Beclin-1, p62, LC3 II/I,P-AMPK and P-ULK1 in HT29 cells pretreated with varied concentrations of curcumin for 24 h and then 20 μM of 5-Fu for 24 h. *, *p* < 0.05 and **, *p* < 0.01 and ***, *p* < 0.001 compared to the placebo (0 μM curcumin) cell group. (PDF 218 kb)

Additional file 5: Figure S5. Immunofluorescent images of HCT116 cells. DAPI staining (blue) indicates nucleus, TUNEL staining (green) indicates apoptosis. (PDF 142 kb)

## Abbreviations

5-Fu + Cur: Co-treatment with 5-Fu and curcumin
5-Fu: 5-Fluorouracil
Cur: Curcumin
pre-5-Fu: Pretreatment with 5-Fu followed by curcumin
pre-Cur: Pretreatment with curcumin followed by 5-Fu
